# Invasive Mucormycosis – An Enigma

**DOI:** 10.7759/cureus.20475

**Published:** 2021-12-17

**Authors:** Anil Prasad, Minakshi Mishra, Kaushik Saha

**Affiliations:** 1 Pathology, Tata Main Hospital, Jamshedpur, IND

**Keywords:** spores, non-septate, immunocompromised, diabetes, invasive

## Abstract

Mucormycosis is an emerging infection in the present post-COVID-19 era, associated with high morbidity and mortality. We are reporting an interesting case of invasive rhino-orbital-cerebral mucormycosis in a 65-year-old female who presented with left nasal and orbital swelling after COVID-19 infection associated with uncontrolled diabetes mellitus. Histopathological and microbiology examination favored mucormycosis. Finally, endoscopic debridement of the lesion was done with left orbital exenteration. The patient at present is clinically stable. As these cases have been seen in many suspected and confirmed COVID-19 cases, early diagnosis and treatment will salvage the patient.

## Introduction

Rhino-orbital-cerebral mucormycosis (ROCM) is a rare, invasive, and rapidly progressive fungal infection affecting the nose and paranasal sinuses that may often extend to orbit, brain, and palate. Being lethal in immunocompromised, like those with diabetes, it needs an early therapeutic approach, including aggressive surgical and medical interventions. ROCM remains a life-threatening infection with a poor prognosis. It is also diagnosed in a few cases after post-mortem [1,2]. The disease is caused by fungi Mucor, Order Mucorales. Its prevalence in India is 0.14/1000 population [3].

Mucormycosis is most commonly associated with diabetes mellitus as a risk factor in India [4]. Type 2 diabetes has a high prevalence rate in India (8.9% of adults) [5]. Patients with uncontrolled diabetes and immunocompromised status have a high incidence of orbital and cerebral involvement. Due to high severity, patients may die despite receiving therapy [6-11].

## Case presentation

A 65-year-old female, who had a COVID-19 infection 2 weeks ago, came to the outpatient department with complaints of swelling on the left side of the nose and eye for 7 days. 

On clinical examination, there was mucopurulent discharge seen from the left nasal cavity, necrosed middle turbinate, proptosis of the eye with purulent discharge (Figure 1), and loss of vision and eye movements.

**Figure 1:** Clinical image showing periorbital involvement.

The routine blood investigations sent on admission were collected (Table 1) and the sugar profile test was grossly deranged.

**Table 1:** Initial lab investigations of the patient. TLC, total leukocyte count.

Parameter	Patient's value	Normal range
Hemoglobin (g/dl)	9.4	11.5-16.5
TLC (cells per mm^3^)	13,900	4,000-11,000
Platelet (cells per mm^3^)	1,52,000	150,000-450,000
Random blood glucose (mg/dl)	392	110-145
Glycosylated hemoglobin (%)	12.5	4-6
Serum creatinine (mg/dl)	1.3	0.5-1.5

Radiological examinations and magnetic resonance imaging (MRI) (Figure 2) show peripheral enhancing soft tissue swelling in the left orbital region with extension to the left cavernous sinus, pterygopalatine fossa.

**Figure 2:** A and B, Radiological images (cranial MRI) of invasive rhino-oculo-cerebral mucormycosis. A: Axial FLAIR, soft tissue swelling in the left orbital region (arrow indicates extension to the left cavernous sinus). B: Axial T2, further deeper extension of the lesion (arrow indicates left pterygopalatine fossa involvement). MRI, magnetic resonance imaging; FLAIR, fluid-attenuated inversion recovery.

Incisional biopsy was taken from the left nasal cavity and middle turbinate. Histopathological examination shows grossly single whitish tissue measuring 2.5 × 0.8 × 0.6 cm.

Microscopic examination with routine hematoxylin & eosin (Figure 3) showed abundant necrosis along with chronic inflammatory cells. Plenty of right-angle branching, broad nonseptate hyphae and spores were seen suggesting fungal infection of mucormycosis. 

**Figure 3:** Microphotograph showing broad-angled aseptate fungal hyphae (40×, hematoxylin and eosin).

Special stains with periodic acid-Schiff (PAS) highlighted fungal hyphae (Figure 4), confirming the diagnosis.

**Figure 4:** Microphotograph showing periodic acid-Schiff stain-positive eosinophilic fungal hyphae (40×).

Finally, endoscopic debridement of the lesion was done with left orbital exenteration. The patient was given systemic anti-fungal treatment liposomal IV amphotericin and other broad-spectrum antibiotics. She showed good clinical improvement.

## Discussion

India reported COVID-19-induced mucormycosis in a vast majority of different regions. The cases already started increasing before the pandemic and reached its peak during a pandemic. India has a large number of diabetic patients and nearly 70% of these have uncontrolled diabetes. High environmental temperatures with tropical and subtropical humid climates also contribute to a high prevalence of the disease.

After COVID-19 infection, mucormycosis is a serious health issue. It is an opportunistic fungal disease seen in patients with uncontrolled diabetes and COVID-19 patients on long-term steroids treatment, solid organ transplants, and severe neutropenia. The most common species isolated was the Rhizopus species, with an overall mortality of 46% [12].

Mucormycosis in healthy individuals are very rare. Most people develop this infection by breathing mold spores. Preexisting diabetes, use of immunosuppressive therapy, known previous respiratory pathology, hospital-acquired infections, etc. and a complex interplay of all factors have a significant impact on patient morbidity and mortality. Diabetes mellitus was a common risk factor in most of the patients.

It can also affect the brain, heart, spleen, kidney, lung, and other organs. Generally, these infections have five presentations: rhino-cerebellar, pulmonary, cutaneous, gastrointestinal, and disseminated [13].

ROCM is a fulminant infection of the nasal cavity, paranasal sinuses, and orbital soft tissue and finally affects the central nervous system. Invasive and noninvasive are two basic types of fungal infections. Microscopically angioinvasion is an important hallmark of mucormycosis infections with resultant vessel thrombosis and tissue necrosis. Perineural/neural invasion may be present in a few cases. Mucorales possess unique virulence traits, which help the organism to exploit the state of immunosuppression and physiologic impairment of phagocytosis seen in this subset of patients [14]. Granulomatous inflammation with multinucleate giant cells, the predominance of lymphocytic cells, widespread necrosis, and degenerated tissue are other characteristic features along with broad aseptate eosinophilic hyphae. The density of fungal organisms is higher in the necrotic tissue. A good sampling of necrotic tissue is highly suggested for the diagnosis of fungal elements. Fine-needle aspiration cytology, squash/imprint, or scrape smear where available often helps in the identification of the fungal organism.

The early timely intervention of surgery and antifungal therapy has a key role in the treatment of COVID-19-associated mucormycosis. Most of the cases need sinonasal surgical debridements [15]. It is also associated with higher patient survival with reduced disease morbidity and mortality.

A high index of clinical suspicion, low threshold for diagnosis in patients with risk factors, neuroimaging, histopathological examination, fungal culture, and polymerase chain reaction are very important for early diagnosis. Special stains like PAS, Grocott methenamine silver, and Ziehl-Neelsen stain (in case of granulomatous inflammation) help to demarcate the fungal elements in the tissue.

## Conclusions

This case illustrates that invasive mucormycosis is a rare opportunistic infection occurring in COVID-19 patients with high-dose steroids, uncontrolled diabetes, or on immunosuppressive therapy and associated with high morbidity and mortality.

Histopathological confirmation and fungal culture are important for confirmation of diagnosis. Strong clinical suspicion, early extensive investigations, multidisciplinary approach, and management can help us save these types of fatal cases.
